The article "Platelet-To-Lymphocyte and Neutrophil-To-Lymphocyte Ratios Predict Intestinal Injury in Male Heroin Addicts" was retracted in 2023. Reasons: unreliable results or conclusions; concerns about the data; concerns about the peer review; concerns about the citations.

# Platelet-To-Lymphocyte and Neutrophil-To-Lymphocyte Ratios Predict Intestinal Injury in Male Heroin Addicts

**DOI:** 10.1155/2022/2195330

**Published:** 2022-07-16

**Authors:** Xinfeng Zhang, Xiaoli Zhang, Huayou Luo, Ruo Shu, Li Guo, Jinghong Zhou, Bowen Tan, Xiao Guo, Yuhan Wang, Yan Tian

**Affiliations:** Department of Gastrointestinal and Hernia Surgery, The First Affiliated Hospital of Kunming Medical University, China Kunming, Yunnan 650032

## Abstract

**Objective:**

To explore the potential link between gut damage and proinflammatory cytokines in heroin-dependent patients.

**Methods:**

We retrospectively analyzed and compared partial blood counts and biomarkers of intestinal injury and their potential correlations in 38 male heroin abuse patients and 29 healthy male participants. In addition, we compared and assessed proinflammatory cytokines and immune cells in 10 heroin abuse patients and 10 healthy participants.

**Results:**

Neutrophil counts, platelets/lymphocytes (PLR), neutrophils/lymphocytes (NLR), gut injury biomarkers, and proinflammatory cytokines, CD19+B in patients compared with healthy subjects' cells increased significantly. The number of lymphocytes, CD3 CD4 T cells, and CD3 CD8 T cells decreased in patients compared to healthy individuals. When distinguishing between heroin addicts and healthy people, ROC/AUC analysis showed that a cutoff of 142.42 for PLR and 2.18 for NLR yielded a sensitivity of 65% and 85% and a specificity of 96.5% and 89.7%, respectively (*p* = 0.001, *p* < 0.001). For predicting intestinal injury, ROC/AUC analysis showed that a cutoff of 135.7 for PLR and 0.15 for NLR yielded a sensitivity of 52% and 60% and a specificity of 82% and 86.4%, respectively (*p* = 0.003, *p* = 0.009). Male heroin addicts are subject to intestinal injury and present with increased proinflammatory cytokine levels.

**Conclusion:**

NLR and PLR are possible indirect biomarkers for heroin dependence based on intestinal injury.

## 1. Introduction

Heroin and related use disorders continued to increase in U.S. adult men and women from 2002 to 2018 [1, 2]. Heroin-related deaths increased from 13,000 to 62,000 per year between 2002 and 2018 and continues to increase [3]. In addition to regulating metabolism, the microbiome-gut-brain axis also plays a vital role in regulating behavior [4]. Heroin abuse affects the brain via central dopamine-reward pathways [5]. In addition, compared with healthy subjects, intestinal microbiota changes in substance use disorders [6]. Harmful bacteria increase the production of inflammatory cytokines, triggering infiltration of inflammatory cells (such as neutrophils), leading to tissue damage and necrosis [7, 8]. For example, gram-negative bacterial endotoxin (BT) is a potent activator of the host immune response and can activate the transcription factor nuclear factor kappa B [9, 10], which leads to the production of cytokines [11, 12]. The epithelial cells, mucus, mucins, and antibacterial proteins produced by the intestinal epithelium establish physical and biochemical barriers to protect the intestines from infectious agents [13]. While it has been reported that intestinal injury and intestinal flora changes are caused by alcohol [14–16] and methamphetamine dependence [17], there are currently no studies investigating intestinal injury in heroin addicts. Existing biomarker tests, which are traditionally used to assess the intestinal injury, namely, diamine oxidase (DAO), D-lactic acid (DLC), and bacterial endotoxin (BT), are expensive, complicated, and unnecessary for every substance abuser. There is a need for a simpler and cheaper way to screen whether the heroin addicts have intestinal injury. Here, we explore whether heroin abuse causes intestinal damage and the relationship between intestinal damage and proinflammatory cytokines. In addition, we examined whether the neutrophil-to-lymphocyte ratio (NLR) and platelet-to-lymphocyte ratio (PLR) are related to intestinal injury in heroin addicts.

The article "Platelet-To-Lymphocyte and Neutrophil-To-Lymphocyte Ratios Predict Intestinal Injury in Male Heroin Addicts" was retracted in 2023. Reasons: unreliable results or conclusions; concerns about the data; concerns about the peer review; concerns about the citations.

## 2. Methods

### 2.1. Subjects

The following are the inclusion criteria: (1) male heroin patients over 18; (2) complete patient data and history; (3) the last heroin abuse which was within two weeks; (4) without digestive tract diseases; (5) without common cold, fever, pain, active infections, and various diseases that may cause abnormal blood cell counts; and (6) patients which are heroin-addicted and develop intestinal damage.

The following are the exclusion criteria: participants with a history of diabetes mellitus or other chronic wasting diseases, who were HIV-positive, were HCV-positive, or had any severe psychosis and bleeding disorders, or were taking anticoagulant drugs. Exclude patients with incomplete clinical information.

Thirty-eight male heroin abuse patients and 29 male health participants from the First Affiliated Hospital of Yunnan and Kunming Medical University were included in the study. The 29 control male patients were healthy blood donors without any history of drug abuse, and all met the inclusion criteria except the second criterion. All study subjects provided written informed consent to the study protocol, which was approved by the Ethics Committee of Yunnan and the First Affiliated Hospital of Kunming Medical University, Kunming, China. No patients dropped out of the study.

### 2.2. Data Collection

To calculate the NLR, divide the absolute neutrophil count by the absolute lymphocyte count. To calculate the PLR, divide the absolute platelet count by the absolute lymphocyte count [18]. To calculate the PLR, divide the absolute platelet count by the absolute lymphocyte count [19]. Data on patient history were collected from our early questionnaire records retrospectively. At the same time, blood cell counts, proinflammatory cytokines, and partial immune cells were extracted from the medical records. All blood samples were collected within two weeks, and gut injury biomarker data were extracted for each patient during the same year.

The article "Platelet-To-Lymphocyte and Neutrophil-To-Lymphocyte Ratios Predict Intestinal Injury in Male Heroin Addicts" was retracted in 2023. Reasons: unreliable results or conclusions; concerns about the data; concerns about the peer review; concerns about the citations.

### 2.3. Statistical Analysis

Statistical analysis was conducted using IBM SPSS version 21 (IBM Corporation, Armonk, NY, USA). Student's *t*-test or Mann–Whitney *U* test was used to compare two independent groups according to distribution status. Variance (ANOVA) was used to test the difference between the mean values of some parameters in the two groups. We presented correlations between two variables using Spearman's or Pearson's correlation coefficient. Finally, we analyzed the receiver operating characteristic (ROC) curve to determine the discrimination values of NLR and PLR for study subjects with or without intestinal injury. A value of *p* < 0.05 was considered statistically significant.

## 3. Results

### 3.1. Patient Characteristics

The characteristics of the 67 participants are presented in Table 1. No significant differences were observed between the age of the two groups (patient group: 36.50 ± 7.83 years; control group: 33.03 ± 12.04 years). However, parameters other than age were statistically significant between the two groups. Table 1 shows that the mean intestinal injury biomarkers, including DAO, DLC, and BT, were significantly higher in the patient group (DAO: 12.28 U/L, DLC: 17.27 mg/L, and BT: 20.19 U/L) than those in the control group (DAO: 7.94 U/L, DLC: 12.67 mg/L, and BT: 17.03 U/L). The mean PLR was significantly higher in subjects in the patient group (PLR: 161.54) than in subjects in the control group (PLR: 103.30); the mean neutrophil count and NLR were significantly higher in patients than in control subjects. Inversely, lymphocyte count was significantly higher in control subjects than in patients. However, there was no significant difference in platelets between the two groups.

### 3.2. Correlation Analysis

Table 2 shows the comparison of laboratory data and PLR or NLR in heroin addicts. There was a clear correlation between the DLC, NLR, and PLR (DLC and PLR, correlation coefficient: 0.431, *p* = 0.007; NLR and PLR, correlation coefficient: 0.717, *p* = 0.002), but there were no significant differences between NLR and intestinal injury biomarkers (DAO and NLR, correlation coefficient: -0.024, *p* = 0.888; DLC and NLR, correlation coefficient: 0.164, *p* = 0.327; BT and NLR, correlation coefficient: 0.007, *p* = 0.967). In addition, DAO or BT also had no significant correlation with PLR (DAO and PLR, correlation coefficient: -0.124, *p* = 0.397; BT and PLR, correlation coefficient: 0.205, *p* = 0.217). A positive correlation was observed between NLR and PLR, and between DLC and PLR.

The article "Platelet-To-Lymphocyte and Neutrophil-To-Lymphocyte Ratios Predict Intestinal Injury in Male Heroin Addicts" was retracted in 2023. Reasons: unreliable results or conclusions; concerns about the data; concerns about the peer review; concerns about the citations.

### 3.3. ROC Curve for Diagnosing the Intestinal Injury

Based on ROC curve analysis, the area under the curve (AUC) was 0.795 (95% CI: 0.653 to 0.936, *p* = 0.001) with a sensitivity of 65% and a specificity of 96.6% with a cutoff of 142.42 for PLR, and the AUC was 0.92 (95% CI: 0.83 to 1, *p* < 0.001) with a sensitivity of 85% and a specificity of 89.7% with a cutoff of 2.18 for NLR, indicating that NLR was superior to PLR as a biomarker to distinguish between heroin addicts and healthy people (Figure 1(a)). For predicting intestinal injury in heroin addicts, ROC/AUC analysis showed a sensitivity of 97% and a specificity of 50% when a cutoff value of 84.79 was used for PLR (*p* = 0.05) (Figure 1(b)). The ideal NLR cutoff value of 2.21 had 87.5% sensitivity and 50% specificity (*p* = 0.20). Considering the small sample size and intestinal injury among healthy individuals, we also included data from healthy individuals. For predicting intestinal injury in all participants, ROC/AUC analysis showed a sensitivity of 52% and a specificity of 82% when a cutoff value of 135.7 was used for PLR (*p* = 0.003) (Figure 1(c)). The ideal NLR cutoff value of 2.51 had 60% sensitivity and 86.4% specificity (*p* = 0.009).

### 3.4. Inflammatory Cytokines and Immune Cells

Focusing on the changes in blood cell counts, we started looking for mechanisms that may cause intestinal injury, so we focused on changes in cytokines and immune cells in the two groups. We selected only 10 individuals per group for this study. Certain cytokines, including IFN-*γ* (patient group: 9.53 ± 10.54 versus control group: 1.99 ± 2.70, *p* = 0.0004), TNF-*α* (patient group: 8.94 ± 2.42 versus control group: 4.36 ± 3.58, *p* = 0.0035), IL-6 (patient group: 18.16 ± 22.17 versus control group: 0.95 ± 0.84, *p* = 0.0246), IL-8 (patient group: 21.89 ± 10.45 versus control group: 6.36 ± 1.67, *p* < 0.0001), and IL-12 (patient group: 1.83 ± 0.62 versus control group: 1.19 ± 0.29, *p* = 0.0087), were significantly different between the two groups (Figures 2(a)–2(g)). IFN-*α* (patient group: 20.81 ± 37.50 versus control group: 1.87 ± 1.40) and IL-1*β* (patient group: 19.23 ± 18.09 versus control group: 12.01 ± 1.47) were not significantly different between the two groups, but we can see that the levels are slightly higher in heroin addicts than in healthy controls. Certain immune cells, such as CD3+CD4+ T cells (patient group: 18.31 ± 3.96 versus control group: 22.97 ± 1.63, *p* = 0.0029) and CD19+ B cells (patient group: 24.75 ± 5.09 versus control group: 16.67 ± 1.98*p* = 0.0173), were significantly different between the two groups (Figures 3(a) and 3(b)). The amount of CD3+CD8+ T cells (patient group: 18.71 ± 3.96 versus control group: 22.47 ± 5.64, *p* = 0.0915) and macrophage cells (patient group: 1.19 ± 1.18 versus control group: 0.39 ± 0.21*p* = 0.0504) was not significantly different between individuals in the two groups (Figures 3(c) and 3(d)).

The article "Platelet-To-Lymphocyte and Neutrophil-To-Lymphocyte Ratios Predict Intestinal Injury in Male Heroin Addicts" was retracted in 2023. Reasons: unreliable results or conclusions; concerns about the data; concerns about the peer review; concerns about the citations.

## 4. Discussion

The initial objective of the study was to identify intestinal injury-induced bacterial translocation and endotoxemia in heroin addicts. DAO, DLC, and BT serum concentrations are traditionally used to evaluate enterocytic damage and dysfunction. Intestinal injury is strongly correlated to damage caused by inflammation, and the NLR and PLR are reportedly better inflammatory indicators than WBC count [20]. The results of our study indicate that the NLR and PLR can be used to evaluate intestinal injury in heroin addicts and healthy individuals. In addition, there were significant differences in the levels of certain cytokines and immune cells between the two groups, which may be related to intestinal damage.

Recent studies have demonstrated that elevated PLR and NLR can serve as biomarkers for disease status in cancer. According to Feng et al.'s study [21], a PLR test can be used to determine the diagnosis and prognosis of patients with esophageal squamous cell carcinoma [21]. The NLR is also a promising marker in solid tumors, and a meta-analysis [22] showed that a high NLR is associated with overall adverse survival in patients with various solid tumors, such as gastroesophageal carcinoma hepatocellular carcinoma, and breast cancer [22]. Moreover, the NLR and PLR are widely used to assess different inflammatory diseases, such as liver fibrosis and cirrhosis [23], thyroid ophthalmopathy [24], Behçet's disease [25], and acute coronary syndrome [26]. Based on previous studies, we explored whether the PLR and NLR are closely related to intestinal injury in heroin addicts.

Current research on heroin addicts focuses on finding alternative treatments, addiction mechanisms, and alleviating withdrawal reactions, while less research on gut damage is currently available. Our study showed that traditional intestinal injury biomarkers (serum concentrations of DAO, DLC, and BT), PLR, and NLR have significant differences between healthy subjects and heroin abusers. DAO is a catabolic enzyme that is typically present in the intestinal mucosa and villi, and its serum concentration can reliably reflect the integrity and maturity of the intestinal mucosa [27]. Human Bacteroides fragilis mainly produce DLC under anaerobic growth conditions, and an increased serum concentration indicates that intestinal wall permeability is increased [28, 29]. A variety of endotoxins can be found on gram-negative bacteria's surfaces, and they are amphiphilic macromolecules and increased serum concentrations indicate bacterial translocation from the gut [30]. We believe that heroin induces significant increases in apoptosis in the intestine by direct or indirect means. Intestinal mucosal damage includes decreasing crypt proliferation, crypt number, and villus height. The gastrointestinal tract harbors a vast population of commensal bacteria [31]. We speculate that the NLR and PLR can not only distinguish between heroin addicts and healthy people but can also identify intestinal damage in heroin addicts. Although our results show no significant difference in finding intestinal injuries among heroin addicts using the NLR and PLR, these markers were significantly different when examining all study participants. Nevertheless, the current efforts will undoubtedly prove invaluable.

The article "Platelet-To-Lymphocyte and Neutrophil-To-Lymphocyte Ratios Predict Intestinal Injury in Male Heroin Addicts" was retracted in 2023. Reasons: unreliable results or conclusions; concerns about the data; concerns about the peer review; concerns about the citations.

Previous studies have shown that inflammatory cytokines and immune cells are involved in intestinal damage. Inflammatory cytokines can promote bacterial association with the epithelium or might react with harmful bacteria to enhance their invasive characteristics [32, 33]. Animal experiments have shown that high levels of TNF-*α*, IL-1*β*, IL-8, IL-12, and IL-6 can lead to intestinal damage [7, 34, 35]. T cell-derived IFN-*γ* promotes intestinal stem cell apoptosis and pathology [36, 37]. Likewise, B cells also contribute to intestinal damage [38]. Moreover, it is well known that neutrophil reactive oxygen species production also induces intestinal damage [39]. We hypothesize that our results show lymphocytes performed poorly in heroin addicts, mainly due to a high consumption status.

This study also has some shortcomings. These findings may be somewhat limited due to the lack of available data for heroin addicts, and a larger study cohort would provide more accurate results. Another limitation is that we did not observe the physical intestinal injury in heroin addicts, and no relevant animal or cell experiments exist to support our study. The findings of this study have important implications for using the PLR and NLR as intestinal injury biomarkers in heroin addicts. This approach is advantageous in that it is a simple, cost-effective strategy to explore intestinal injury. Further research is necessary to explore the reliability of using the PLR and NLR, and future *in vitro* and *in vivo* studies are required to substantiate the findings of this study.

The article "Platelet-To-Lymphocyte and Neutrophil-To-Lymphocyte Ratios Predict Intestinal Injury in Male Heroin Addicts" was retracted in 2023. Reasons: unreliable results or conclusions; concerns about the data; concerns about the peer review; concerns about the citations.

## 5. Conclusion

Intestinal damage in heroin addicts may be associated with translocation-induced production of proinflammatory cytokines by translocation of bacteria and their products. PLR and NLR have potential clinical applications as biomarkers for intestinal injury.

## Figures and Tables

**Figure 1:** ROC curve for diagnosing the intestinal injury.

**Figure 2:** Inflammatory cytokine level.

**Figure 3:** Percentage of immune cells.

**Table 1:** The characteristics of the study participants.

	Heroin abusers	Health subjects	*p* value
	(*n* = 38)	(*n* = 29)	
Age (years)	36.50 ± 7.83	33.03 ± 12.04	0.159
DAO (U/L)	12.28 ± 5.05	7.94 ± 2.61	^∗∗∗^
DLC (mg/L)	17.27 ± 4.05	12.69 ± 5.84	^∗∗∗^
BT (U/L)	20.19 ± 4.08	17.03 ± 3.61	^∗∗^
N (10^9^/L)	6.09 ± 2.01	3.51 ± 1.28	^∗∗∗^
L (10^9^/L)	1.68 ± 0.60	2.39 ± 0.54	^∗∗∗^
P (10^9^/L)	246.84 ± 64.77	234.66 ± 39.34	0.374
PLR	161.54 ± 62.57	103.30 ± 29.57	^∗∗∗^
NLR	4.11 ± 2.29	1.5 ± 0.50	^∗∗∗^

^∗∗∗^ *p* < 0.001. ^∗∗^*p* < 0.01. Values are the mean ± SD. DAO: diamine oxidase; DLC: D-lactic acid; BT: bacterial endotoxin; N: neutrophil; L: lymphocyte; P: platelets; PLR: platelet-to-lymphocyte ratio; NLR: neutrophil-to-lymphocyte ratio.

**Table 2:** Correlation analysis between PLR/NLR and intestinal injury biomarkers in the patient group.

	Variable	*n*	Correlation coefficient	Significance (two-tailed)
PLR	DAO	38	-0.142	0.397
	DLC	38	0.431^a^	0.007
	BT	38	0.205	0.217
	NLR	38	0.717^a^	0.002
NLR	DAO	38	-0.024	0.888
	DLC	38	0.164	0.327
	BT	38	0.007	0.967

^a^ *p* < 0.01 (two-tailed) was considered statistically significant. DAO: diamine oxidase; DLC: D-lactic acid; BT: bacterial endotoxin.

## Data Availability

The datasets used and analyzed during the current study are available from the corresponding author upon reasonable request.
